The article "Community Construction and Development Path Analysis of Ecological Environment-Friendly Elderly Care Service" was published in 2023. Journal: J Environ Public Health.

# Community Construction and Development Path Analysis of Ecological Environment-Friendly Elderly Care Service

**DOI:** 10.1155/2023/1982767

**Published:** 2023-01-31

**Authors:** Jie Guo, Wenjie Li, Wenhao Ling

**Affiliations:** ^1^Institute of Administration Study, Henan University, Kaifeng, Henan, China; ^2^School of Public Administration, North China University of Water Resources and Electric Power, Zhengzhou, Henan, China; ^3^Institute of Social Governance Research Center, Henan University, Kaifeng, Henan, China

## Abstract

As a new pension model, ecological pension is an important choice to relieve the pressure of population aging in China. This paper reviews the relevant literature on the integrated development of the ecological pension industry and rural revitalization in recent years and points out that the researchers have determined the model of the ecological pension industry, the path of rural revitalization, the comprehensive development of organic pension industry, and rural revitalization and the problems they face. Some results have been achieved. However, there is still a lot of research space for the integrated development of the ecological pension industry and rural revitalization, especially to establish a perfect index system of the ecological pension industry, the measurement standard of rural revitalization, and the theoretical basis and mechanism of integrated development. Regional cooperative symbiosis is based on industrial symbiosis. In terms of research methods, attention should be paid to the combination of theoretical analysis and empirical research, to the further development of this field, and to achieve remarkable results. In the process of social and economic development, the rural ecology can be built by solving the problems of the elderly, accurately reducing rural poverty, and protecting the environment. The healthy elderly care tourism destination has realized the integrated development of rural tourism, ecological health tourism, and elderly care tourism. Taking Chang'an District of Xi'an as an example, the advantages of the district in geographical location, climate, environment, tourism resource health, as well as the constraints in the system, talent, policy, and system are demonstrated, and the corresponding countermeasures are put forward.

## 1. Introduction

With the acceleration of population aging, the reduction of family size, the mobility of the labor force, and the weakening of family relations, the traditional home care model can no longer meet the needs of the elderly. While home care is unsustainable, scientists note that providing Jolo services is an important trend to address the challenges of an aging population. Local governments actively promote the nonprofit model, and they also encounter many problems and challenges in the process of development. In particular, the imbalance and shortage of welfare benefits, resource allocation, and regional differences are significant. The unbalanced and insufficient development of nonprofit services at home and abroad hides the core attribute of public goods and the core value of fairness and accessibility.

People need more qualities and happiness in their later years. On August 23, 2020, the Ministry of Civil Affairs announced its latest forecast. During the four-year and five-year plan (2021–2025), China's elderly population (over 60 years old) has exceeded 300 million, leading to mild to moderate aging. In five to 10 years, China's first parents have entered the elderly stage, and the national pension institutions are a direct challenge to the challenges and tests. With the rapid development of China's pension industry, new models, new technologies, and new businesses are constantly driving new changes. More and more older people want to enrich their lives and improve their health. In this context, the rural ecological industry has gradually become a major development direction in the new era. With the development of information technology, community information platforms and sensor network systems of pension organizations constantly appearing, making the ecological pension industry more intelligent and scientific. In recent years, pension organizations have failed to meet the needs of the elderly [1]. With the planning and construction of many suburban gardens, farms, farms, and rural farms, the principle of development centered on the quality of life for the elderly was further implemented, as shown in Table 1.

## 2. State of the Art

### 2.1. The Urgent Need for Pension Services

As shown in Table 2, ecotourism is a way of tourism appearing along with the aging of the population and the improvement of the subhealth level. This study aims to develop in-depth tourism experiences based on natural and cultural environments. Senior travel is essentially a vacation for the elderly. That is to say, the elderly leave the original residential area and travel to a good destination for half a year, engaged in leisure, vacation, sightseeing, leisure, and other activities. Elderly tourism is a new integration of the elderly and tourism, which can not only improve the quality of life of the elderly but also reduce the social pressure on the elderly, alleviate the problem of seasonal tourism facilities in tourist destinations, and promote the development of tourism [2].

China is entering an aging society. According to the latest statistics, 17.9 percent of China's population is over 60. Elderly care is an important issue in Japan. As China's national income grows, tourism has become a new fashion for the elderly. Especially when the scenery is beautiful and the air is fresh and back to the comfortable rural sightseeing place, the elderly can meet their sightseeing needs and jro needs. Therefore, for the healthy elderly people with high economic burdens, it is a new trend to receive elderly care services in rural ecotourism.

#### 2.1.1. Government-Led, Multisubject System

For the elderly, the government only builds the infrastructure for the elderly. Public finance and society raise funds, invest in infrastructure, and provide pension services. Under the active guidance of various social groups and organizations, the government has formed a nonprofit network composed of companies and volunteer service organizations to significantly reduce the pressure on the government. At the same time, the government will start by providing complex and specific services, better playing the leading role of the government, and using various social resources to improve the operational efficiency of [3], as shown in Table 3.

#### 2.1.2. Perfect Infrastructure for the Elderly

As shown in Figure 1, it is said to be one of the most suitable countries for elderly people in the world, with perfect social security facilities. In March 2016, the government launched the “Happy Aging of the Elderly” program to care for the elderly in the construction of various communities. The first floor has plenty of space for community organizations, kindergartens, education centers, community hospitals, senior citizens' activities, and markets convenient transportation. The bus station has a special corridor where old people do not slip in the weather. The city also has daycare centers and rehabilitation centers, providing services to elderly families with children. However, communities with special needs offer a variety of white-and-white meetings and activities to enrich the lives of older people. These measurements are very fine. However, from the interest in this daily life, older people in Singapore can enjoy a relatively rich life in later life and there is no need to stay at home and live a good life [4].

#### 2.1.3. Relevant Laws Are Very Sound

He was a pioneer in protecting the rights of the elderly and was the first Frenchman to support his parents. In 1944, the government passed several laws to support parents and established strict work evaluation and supervision. All indicators have certain quantitative rules, which can avoid subjective intolerance. The establishment of the Standardization Council for the Elderly Elderly emphasizes not only professional pension laws but also the standardization of pension services. To ensure the quality of geriatric care, Singapore has enacted a series of standardized laws such as the Geriatric Care Regulations and the Geriatric Care Regulations. Thus, the assessment and monitoring of urban Yoro services can be based on criteria that support the quality of services and effective monitoring.

### 2.2. Aging of the Pension Service System and Incompatibility to the Social Status Quo

In 2018, the following comments were made: “good leisure agriculture, rural tourism projects, and opinions on building a reasonable form of industry.” Further emphasis on the overall direction of pension development and rural development. China is experiencing a serious wave of aging, and the number of older people is growing at an unprecedented rate. Existing pension organizations cannot meet people's actual expectations about the quantity and quality of noodles [5]. The disadvantages of the traditional pension model are becoming increasingly obvious. With the significant improvement of people's living standards, the healthy and ecological pension model is an important trend in the development of the pension industry and also the desire of the elderly. Due to the above-given social development background, some natural and ecological resources in excellent rural areas provide more development opportunities. It makes full use of its unique ecological resources, develops the ecological criticism industry, and combines the ecological agriculture with the organic agriculture. The industry serves as a leisure tourism, as shown in Figure 2.

In order to promote the rapid development of the rural economy and the rapid realization of rural development, the literature research integrating ecological luo industry with rural development can provide a reference for the research in related fields. Local governments actively promote the nonprofit pension model, and they also encounter many problems and challenges in the process of development, as shown in Table 4. In particular, the imbalance and shortage of pension benefits, unbalanced resource allocation, and regional differences are significant. The imbalance and inadequacy of the development of residential procurement violate the property of public goods, namely, “benefit sharing” and “fair and reasonable.” This is consistent with this point in the 19th report. The National Congress of the Communist Party of China put forward the goal of balancing basic public services in principle [6].

### 2.3. Based on the Ecological Environment-Friendly Elderly Care Service Community

#### 2.3.1. Eco-Environment-Friendly Community-Based Elderly Care Services

The suburban model of the suburban ecological pastoral area is developed, and the power of the state, business, society, and individual are integrated, and the suburban resources are integrated. We should pay more attention to pension issues. At the same time, the gradual deepening of population aging and the personalized demand for the elderly have brought new difficulties and challenges to the development of China's pension insurance industry. With the strong support of national policies, in order to reduce the burden of the government, help the elderly, and comfort the children, the ecological rural pension industry has carried out test points nationwide, laying a solid foundation for the further development of the pension industry [7].

#### 2.3.2. The Advantages of Ecological Environment-Friendly Elderly Care Service in the Community

As people's living standards improve, participation in leisure activities (such as abundant crop cultivation and excursions) increases, especially the holidays contributing to the development of the rural Jro model. We have built an ecological industrial chain model in diversified urban and rural areas, reducing the impact of seasonal changes on the industrial development process of the industry, emphasizing its advantages, and gradually becoming the current ideal social development model.

## 3. Methodology

For the age, environment, facilities, and space problems brought about by the operation of the pension model, the state, individuals, and enterprises have carried out in-depth research on the pension problems. In order to promote the rapid construction of scientific and efficient elderly care facilities, the elderly care services can be gradually improved according to the relevant national policies. We constructed an ecological orro model to combine the dominance of industrial space with the master planning [8].

### 3.1. The Realization of Eco-Environment-Friendly Elderly Care Services

We explore the ecological teachings and characteristics of the suburb as a rural ecological frontier. In recent years, the gap in urban development is not only material but also cultural. We should balance the cultural and material differences between urban and rural areas, create a good interactive model, organically integrate local industries, and develop new suburban and rural ecological support. This development not only reflects the whole noodle development of the new company but also reflects people's yearning for a better life in [9].

#### 3.1.1. Design of Community-Based Living Space for Elderly Care Services

Housing design of rural ecosystems plays an important role in the development of pension models, as shown in Table 5. Due to the poor health status of the elderly, the space for social activities gradually shrinks, and the elderly's dependence on and demand for housing gradually increases. Therefore, the design of a rural ecological nursing home is particularly important. In the design of the living space, the housing of the elderly should be close to the ground, and there should be low residential buildings and small high-grade buildings so that the elderly can choose [10] according to their own family conditions and preferences. Room types were also designed for one and multiple rooms. The Housing feature allows you to receive smart services integrated with a nursing home. Living space mainly includes bedroom, kitchen, toilet, and balcony; it is important to have a living room. To avoid cloudy, snowy, rainy weather, and to reduce recreational activities for older people, elderly people tables, chess boards, television, and movies were installed. In addition, the room, kitchen, bathroom, and balcony in the room design should consider the problems of the elderly, such as slow limb movement and inconvenience. In addition, alarm systems must be installed to ensure the safety of the elderly.

#### 3.1.2. Community-Based Outdoor Space Design for Elderly Care Services

The rural elderly environment includes both the indoor environment and the outdoor environment. To provide a quiet and comfortable outdoor environment for the elderly, you will need to design a green outdoor environment and combine it with a natural ecology. In the outdoor road design of eco-villages, it is necessary to link the outdoor activity areas of the elderly with the convenience of the elderly. Rural pension organizations can organize vehicle associations. The ambulance and fire station were installed to connect the elderly road of the village with the city road to avoid road problems and wasting time [11]. Rural elderly care systems should reduce the use of foreign vehicles and domestic vehicles and prevent exhaust pollution from affecting the quality of the elderly. The primary purpose of rural care is to provide a quality living and rest environment for the elderly. As a new Jolo model, we must attach importance to environmental construction. In addition to planting cherry trees and trees, we must also invest in lakes to bring the elderly closer to nature and provide a place for discussion and games to enrich their future lives. Finally, we established a public cultural institution such as the reading room, library, and computer learning center.

### 3.2. Ecological and Environment-Friendly Old-Age Care Model Service Process

How does the new pension model meet the individual needs of different elderly people? This is the direction that every government and NGOs are looking for. In recent years, the combination of medical treatment and nursing care, the concept of intelligent pension, and the emergence of this model have opened up new development goals for the pension business. With the support of the state and municipal governments, the rural pension model is being gradually improved. The Internet, the Internet of Things, and other technologies are combined to create a more scientific and effective space for the elderly.

#### 3.2.1. Service Mode of Combining Medical Care and Nursing Care

The medical service model combines online and offline services to meet the needs of modern elderly health and care services. With the support of national and local policies, it is possible to achieve people's satisfaction and social welfare through social awareness. In the suburbs, communities use information technology, and health and medical information for the elderly is combined with a modern smart hospital [12]. Hospitals can develop detailed treatment plans, medical care, rehabilitation, and health care services according to the health status of the elderly and can promote the “medical bond” for the elderly, as shown in Figure 3. At the same time, rural pension organizations can customize smart bracelets for the elderly to monitor the health conditions in real time, greatly reducing the probability of accidents.

#### 3.2.2. “Nongjiale” Tourism Service Mode

With the rapid economic development, the elderly have placed more and more emphasis on spiritual enjoyment. Sunset ecological leisure industry, especially leisure tourism is a household name. The rural Yoro ecological model is a cultural display place based on the local historical and cultural construction. Through the interpretation of the traditional Chinese culture, we can inherit the history and culture. Combine the development of the local leisure industry with the characteristic economic industry, to form the local characteristic tourism mode, promote the development of the local economy, and reflect the overall service of the industry.

#### 3.2.3. “Farmhouse Music” Catering Service Mode

The construction of the pension model provides a full range of services for the diet and seats of the elderly, adapts to the special dietary materials, meets the needs of the postpartum taste of the elderly, and provides the quality of life for the elderly. An inconvenient old man can order food through a smart machine and taste delicious food, and you do not have to go to a designated location [13].

#### 3.2.4. Education Service Mode for the Elderly

In the process of developing the education model for the elderly, pension organizations can interact with local universities. The regular selection of teachers and students for education and communication not only inherits the spirit of “learning for the elderly” but also increases the enthusiasm of teachers and students to participate in community service activities [14]. Under the guidance of professional knowledge, the rural pension ecological model not only promotes the improvement of the quality of pension but also promotes the innovative development of pension facilities [15].

## 4. Result Analysis and Discussion

### 4.1. Obtained by the Ecological and Environment-Friendly Elderly Care Service Community Merits and Drawbacks: Merits and Faults

As shown in Figure 4, establishing the rural ecological Joloy model can design the planning mechanism for the reemployment of the rural elderly people. These jobs are mainly suitable for older people engaged in professional and nonprofit businesses. They provide the elderly and dynamic people with the opportunity to realize their own value [16]. At the same time, the elderly can use this method to use the waste heat, which is not only conducive to sports but also conducive to the development of the country.

The choice of an ecological model of the pension industry is one of the frontier problems of industrial economic theory research. Carrying out the revitalization work of agriculture, rural areas, and farmers is an important part of the theoretical research of its development. The scientific path of ecological luo industry integration and rural development are concentrated in four aspects. First, we emphasize the interaction, networking, interactivity, and reciprocity of urban and rural communities in the process of rural construction. Mutual benefit and win-win situation of urban and rural residents are promoting the development of rural areas and is regarded as an important condition for sustainable development [17]. Secondly, the service level of rural farmland is generally low, which is quite different from the actual service demand of the modern elderly. Finally, extreme phenomena appear in the process of development and utilization, the public environmental awareness is weak, and the problem of rural environmental pollution is increasingly prominent. The green pension industry is a new form of industry in China, and the rural promotion strategy has been put forward in recent years. Research by local scientists is very limited and is still in the first stage. Although these research puzzles have some reference value to the development of scientists, the concept of the ecological cleaning industry has not been unified. The index system of ancestral industry and rural promotion is not yet clear [18]. Studies on rural areas in economically underdeveloped areas rarely emphasize the concept of industrial symbiosis, but few studies on industrial symbiosis, as shown in Figure 5.

### 4.2. Revelation

#### 4.2.1. Introduce Multiple Subjects and Broaden Investment Channels

In the pension industry, we can not only maintain the sustainable and healthy development of the industry through the power of the government but also introduce social service organizations, companies, and volunteers by integrating social forces. Introducing social groups can strengthen the ability to organize activities and lay the foundation for more social work. The introduction of the company has played an important role in expanding the funding sources, not only reducing the financial pressure of the government but also expanding the company's business, creating a win-win situation [19]. The participation of volunteers will help to create a harmonious atmosphere of social and cultural exchanges and save more funds for infrastructure construction. Based on the Singapore experience, associations, religious organizations and businesses have played a major role in caring for older people. Therefore, we must also play the positive role of all social groups to promote the development of the pension industry.

#### 4.2.2. We Will Accelerate the Formulation of Laws, Regulations, and Standards for Community-Based Eco-Friendly Elderly Care Services

Strengthening the establishment and improvement of relevant laws and regulations, as well as the formulation of industry standards, is crucial for the long-term development of community pension in China. Article 35 of the Law of the People's Republic of China on the Protection of the Rights and Interests of the Elderly stipulates: “develop community services and gradually establish service facilities and networks to meet the needs of the elderly, such as life services, cultural and physical activities, health care, and rehabilitation” but does not explain what and how to do it. According to China's current level of economic development, the unique culture and needs of the elderly, the current situation of the community pension, the responsibility division of the participants in the community pension, the fund source and use of the community pension, Design of the appropriate institutional arrangements clarify the types of community pension institutions, the content, methods and service quality of community pension services, and the working standards of community pension staff; the access and exit mechanism of third-party participation and the content and standards of volunteers' participation in elderly care services have clear and specific provisions on all aspects of urban elderly care services. The healthy, orderly, and rapid development of China's urban old-age service industry cannot be separated from the common role of all aspects[20].

As shown in Figure 6, strengthening the establishment and improvement of relevant laws and regulations and establishing industry standards are the key to the long-term development of community communication in China. According to Article 35 of the People's Law of China on the Protection of the Rights of the People's Republic of China, “it is not clear whether to develop community services for the elderly, to establish services and networks for life services, cultural and sports activities, health and rehabilitation, and what to do and what to do.” According to China's current level of economic development, the unique culture and needs of the elderly, the status of the children in the community, the occupational labor resettlement of each community pension participant, the source and use of the community children fund, the design of the appropriate level arrangement, and the type of the community future fund are clearly defined. Content and conditions of community pension organizations. Community proposition service mode and quality, community pension work standards, the participation and withdrawal mechanism of third parties, and the participation and standard of volunteer service to elderly care service are clear and specific for each side of urban elderly care service, which promotes the healthy development of urban elderly care service. The rapidly developing city and Jro service industry have become an important road for the development of the elderly [21].

#### 4.2.3. Increasing Investment in Infrastructure Construction

Developing family nurseries needs government support. Western countries are very concerned about the investment and construction of pension infrastructure in developing communities. However, around this week, there are many Chinese communities in the area, such as the Urban Health Center, the Masters, the Super Marquette, and other housing services. There were fitness facilities for all community residents, but few facilities specialized in senior activities at the start of construction. China has a large population and many communities, so all the communities directly facing huge financial pressure need substantial financial support to provide pension facilities. Thus, we were able to invest in nursing homes in a larger community and are gradually promoting them across the country [22].

## 5. Conclusion

In recent years, the community of ecological environment-friendly elderly care service has increasingly become the mainstream of elderly care production, and the state strongly supports the development of the elderly care service community. The community can not only let the elderly enjoy the warmth of home but also enjoy the natural ecology and nature, and their children do not have to give up their work to take care of the elderly.

This paper discusses the policy to promote the opening of the sunset farm pension model. The construction of this model has greatly promoted the socio-economic development and improved the quality of life of the elderly. At the same time, due to the joint participation of the society, enterprises, the state, and individuals, the ecological parenting industry has great development potential, which can not only meet the psychological and physiological needs of the elderly but also promote the development and innovation of the ecological parenting industry.

## Figures and Tables

**Figure 1:** Number of aged care institutions.

**Figure 2:** Structure of China's retirement industry.

**Figure 3:** Three dimensions of building a friendly community for the elderly.

**Figure 4:** The development of the structure of China's pension model.

**Figure 5:** Date on the elderly population.

**Figure 6:** Analysis framework.

**Table 1:** Distribution of typical cases of the rural elderly care service innovation mode nationwide.

Area	Province	Amount	Typical case example
East	Hebei province	4	
	Jilin, Guangdong, Hainan, Tianjin	1	
	Heilongjiang province and Liaoning provinces	3	Harbin Pingfang district government and social cooperative “1 + 4” rural mutual assistance pension model
	Jiangsu province and Shandong province	10	Jiangsu Donghai block “three care in one” rural pension model
	Fujian province	22	Quanzhou city, Fujian province, has the “free lunch” platform
	Zhejiang province	6	Zhejiang Tonglu County “home courtyard body micropension institutions construction
	Shanghai municipality	2	
	Beijing municipality	5	
	Anhui province and Hubei province	7	
	Jiangxi province	3	Anhui Shucheng County “one network two raise three services” model

Central section	Henan province	4	Henan Nanyang city extremely poor personnel “four concentration” model
	Hunan province	2	Hunan Shimen County home care service chain operation model
	Shanxi international gong and drum festival	1	
	Chongqing municipality, Yunnan province, Ningxia Hui Autonomous Region, Qinghai province, Gansu province	1	Guangxi Qinzhou city rural “house for pension” model
	Guizhou province, Inner Mongolia autonomous region, Shaanxi province	3	

West	Sichuan province, the New Phrenm Uygur Autonomous region	4	Kunming city, Yunnan rural “to dance old” model
	The Guangxi Zhuang autonomous region	2	Guizhou Tongren city “five type” rural mutual aid happiness hospital
			Sichuan Luzhou Pension Mutual Aid Association model

Amount	Thirty provincial administrative regions	H7	

**Table 2:** Comparison of the three major pillars of pension in China, the United States, and the Netherlands.

Essential information	Classify	Sample number	Proportion (%)
Age	60–69	675	46.1
	70–79	485	33.1
	80 years old and older	305	20.8

Sex	Man	613	41.8
	Woman	852	58.2

Degree of education	The terminally ill	394	26.9
	Primary school and junior high school	739	50.5
	High school and above	331	22.6

Domicile	City	695	47.4
	Rural area	770	52.6

The resident manner	Live with your children	896	61.2
	Do not live with your children	569	38.8

Marital status	Have a spouse	1095	74.7
	Mateless	370	25.3

Level of income	Low income	550	34.5
	Middle income	474	32.4
	High income	486	33.2

The body is frozen	*n* texture	1267	86.5
	Semi-incompetence	122	8.3

Operative mode	Disability	76	5.2
	Retire	1265	86.3
	Endure	200	13.7

Communicate with your children	Frequent communication	545	37.1
	Not often communicate	920	62.9

**Table 3:** Comparison of the three major pillars of pension in China, the United States, and the Netherlands.

Pension assets comparison		The first pillar	The second pillar	The third pillar	Total
China (2019)	Scale (US $1.00 trillion)	1.29	0.40	0.11	1.80
	(%) in the proportion of GDP	9.03	2.82	0.74	12.59

America (2019)	Scale (US $1.00 trillion)	2.72	17.32	12.16	32.20
	For/% of GDP	12.71	80.83	56.76	150.30

Holland (2018)	Scale (US $1.00 trillion)	0.38	0.95	0.57	1.90
	(%) in the proportion of GDP	43.20	108.00	65.30	216.50

**Table 4:** Index system of equalization of community services for home care.

Level 1 indicators	Secondary indicators	Level 3 indicators	Level 3 indicators	The final weight
Accessibility to home care community services	Starting point (1/3)	Availability (1)	Number of community network service personnel addresses (1/6)	1/18
			Number of sites of community network service facilities (1/6)	1/18
			Type of community point service content (1/6)	1/18
			Community door-to-door service personnel count qi (1/6)	1/18
			Community door-to-door service content rush (1/6)	1/18
			Community door-to-door service content rush (1/6)	1/18
	Process (1/3)	Accessibility (1/3)	Distance from home to community service outlets (1/4)	1/36
			Access to community service point (1/4)	1/36
			Cost from home to community services outlets (1/4)	1736
			Waiting time for on-site service by appointment service personnel (1/4)	1/36
		Affordable (1/3)	Price affordability for community life care services (1/5)	1/45
			Price for community medical care services “I burden (1/5)	1/45
			Price Affordable (1/5)	1/45
			Price Affordable services for Xuxu (1/5)	1/45
			Extra burden (1/5)	i/45
		Acceptability (1/3)	Acceptance of the local environment of the community outlets (1/4)	1/36
			Acceptance of community network services (1/4)	1/36
			Community service reservation system availability (1/4)	1/36
			Acceptance of community door-to-door community services (1/4)	1/36
	Result (1/3)	Adaptable (1/3)	Life care services to the community (1/4)	1/12
			Degree of medical care services to the community (1/4)	1/12
			Degree of cultural and entertainment services to the community (1/4)	1/12
			Spiritual comfort services to the community (1/4)	1/12

**Table 5:** Rural ecological pension evaluation index system.

Target layer	Criterion layer R	Index layer C
Ecological pension	Country nature	Air quality condition C11 vegetation coverage condition C12
	Surround ratio	Tourist attraction conditions C13
	Rural foundation	Distance condition from the city of residence condition C14
		Road traffic facilities: C15
		Country Lighting facilities C16
	Facility R2	Network communication facilities C17 hydropower and heating supporting facilities C18
		Sewage treatment facility C19 accommodation conditions C110 diet conditions cm

Evaluation system	Rural pension	Fitness and recreation and leisure conditions C112
	Condition R3	Medical condition C113 quality of care condition C114
	Rural pension	Service price conditions C115
		Harmony degree of villagers C116
		Financial subsidy policy for investment in pension facilities: C117
		Water, electricity and heating cost subsidy policy C118
		Tax relief policy C119
	Policy R4	Financial support policy C120
		Social capital support policy C121 construction land approval policy C122

## Data Availability

The labeled data set used to support the findings of this study is available from the corresponding author upon request.
